# Bilateral Transverse Facial Cleft as an Isolated and Asyndromic Deformity

**DOI:** 10.5005/jp-journals-10005-1062

**Published:** 2010-08-17

**Authors:** SS Ahmed, Afshan Bey, SH Hashmi, Shaista Parveen, Alirza Ghassemi

**Affiliations:** 1 Chairman, Department of Oral and Maxillofacial Surgery, Aligarh Muslim University, Aligarh, Uttar Pradesh, India; 2 Professor, Department of Periodontics and Community Dentistry, Aligarh Muslim University, Aligarh, Uttar Pradesh, India; 3 Professor, Department of Oral and Maxillofacial Surgery, Aligarh Muslim University, Aligarh, Uttar Pradesh, India; 4 Senior Resident, Department of Oral and Maxillofacial Surgery, Aligarh Muslim University, Aligarh, Uttar Pradesh, India; 5 Consultant, Maxillofacial and Plastic and Reconstructive Surgeon, Aachen University Hospital, Pulwaster, Aachen, Germany

**Keywords:** Macrostomia, transverse facial cleft, craniofacial anomaly.

## Abstract

Congenital macrostomia or transverse facial cleft is a rare congenital craniofacial anomaly, which affects the esthetics and functions of oral cavity. It is usually associated with deformities of other structures developed from the first and second branchial arches. Bilateral transverse cleft, occurring alone is uncommon. Since the deformity is rare, its treatment has not been commonly described in the literature. We report a case of congenital bilateral macrostomia as an isolated, asyndromic deformity to add one more case in the literature and surgical technique has been discussed here.

## INTRODUCTION

Transverse facial cleft (Tassier type 7)^1^ or congenital macrostomia is a rare congenital anomaly,^1,2^ which results from failure of the maxillary and mandibular portions of the first brachial arch to unite.^3,4^ These clefts mostly occur as part of syndromes such as facial dysostosis and branchial arch. Thus isolated transverse facial cleft is a rarity.

The estimated occurrence varies from 1 in 100 to 1 in 300 of all facial clefts.^6^ Various etiopathogeneses have been described. At seven weeks of gestation, the lips separate from the alveolar areas with the formations of a vestibule and maxillary and mandibular swellings then merge laterally to form the cheeks. Here incomplete union results in macro-stomia, which is either unilateral or bilateral. According to Mckenzie and Craig.^7^ The defects of the first brachial arch arise from inadequate arterial blood supply occurring during a period of rapid and critical facial growth and development. Various surgical techniques like Z-plasty, W-plasty, triangular flaps and straight line closure have been described in the literature with variable success.

The cutaneous W-plasty proved rewarding in this patient. One case of isolated, bilateral transverse facial cleft is reported. The clinical features and treatment methods are discussed and illustrated.

## CASE REPORT

A 7-year-old male child was referred to the Department of Oral and Maxillofacial Surgery, Dr ZA Dental College, Aligarh Muslim University, Aligarh from primary health care center, Aligarh. The chief complain of the patient was wide mouth and compromised feeding. Child looked thin and was underweight as compare to the children of same age group. He was born prematurely at six months of gestation by cesarean operation. The obstetric history of mother was G_3_P_2_A_o_ (Gravida 3, Para 2, Abortion O). Child had a history of blood transfusion but the parents of the child neither could furnish any documented evidence nor tell the disease for which of blood transfusion was done.

The extraoral examination revealed that the child had a wide mouth. The angles of the mouth were extending posteriorly on either side but not beyond the anterior border of the masseter. The cleft is not beyond the anterior border of masseter was identified by asking the patient to clinch his teeth. Since the muscle is close to skin, it can be easily palpated. When it contracts on clenching, its anterior border stands clearly. Bilaterally, the clefts were lined with skin externally and with buccal mucosa internally. The demarcation between end of the lips and beginning of the defect was noticeable on close observation (Figs 1A and B). Intraoral examination revealed mixed dentition, with normal eruption time and sequence. Orthopantomogram, revealed mild hyperplasia of the mandible. On further local and systemic physical examination no other abnormalities or congenital anomalies were found.

**Figs 1A and B:** Front profile of patient

## TREATMENT

### Surgical Reconstruction of the Defect

The surgical repair of macrostomia bears structural, functional and cosmetic concerns and five goals which have to be achieved, i.e.

1. Formation of symmetric lips and oral commissure.
2. Reconstruction of the orbicularis oris muscle to restore labial function.
3. Reconstruction of the commissures of the mouth with a natural looking contour.
4. Closure of the defect with minimally visible scar.
5. Prevention of future scar contracture with lateral migration of commissures.^8,9^

**Fig. 2:** Postoperative profile after 3 months

We planned W-plasty to achieve these goals in our patient. Our experience is that W-plasty gives better way to achieve cosmetic and functional goals. Prior to intubation the point for new commissure was determined and marked by accurate measurement of two sides (Fig. 3) as well as observation of the point at which texture of the vermilion border changes from normal mucosa to cleft mucosa.^10^

The patient was prepared for surgical repair under general anesthesia and nasoendotracheal intubation, scrubbed and draped as per the standard surgical protocol. 4 cc of 1:200,000 adrenaline with/lignocaine was infiltrated on both sides of the cheek. Incision was given for W-plasty. Along the borders of incision, dissection of subcutaneous tissue was done to explore the fibers of orbicularies oris muscle. The closure of buccal mucosa with overlapping repair of orbicularis oris was done at the level of normal commissures on the contralateral side using 4.0 vicryl suture material. The commissure was closed by fine mattress suture. The buccal muscles were closed directly with 4.0 vicryl sutures. The skin closure was started from the corner of the mouth. The approximation of edges requires perfection to avoid dog-ear without the need for extending the incision or a further Z-plasty in the respective limb of incision. The integrity of muscle fibers and oral sphincter was performed. On one side and reconstruction of the integrity of the oral sphincter was performed. Same procedure was carried on other side; closure was done with 4.0 vicryl and 5.0 monocryl sutures with half round bodied needle. At the end of procedure the skin closure revealed the pattern of W incision (Fig. 4). The postoperative recovery was uneventful. On 3 months follow-up, there was marked improvement in appearance and function (Figs 1A to 2).^3^

**Fig. 3:** Placing of markings before surgery

**Fig. 4:** Immediate postoperative profile

## DISCUSSION

Congenital macrostomia (transverse facial cleft) is a rare, atypical facial cleft that occurs alone or in combination with other anomalies. It is thought to be a part of the manifestations of the hemifacial microstomia, the second most common congenital craniofacial anomaly.^11^ Unilateral cleft is more common than the bilateral. It could vary from mild form with slight widening of mouth, to severe cleft extending back to the ear. However, cases of severe bilateral transverse facial cleft are exceedingly rare.^5^ Malformations of the mandible and/or ear are almost always present.^3^

Various classifications have been given to describe atypical facial cleft but Tessier’s system based on his clinical observation, is most widely accepted.^1^ In Tessier system, clefts are numbered around the orbit from 0 to 14 and clefts # 0 to # 7, depict the facial clefts. The case which we are reporting had bilateral # 7 clefts.

Genetic and environmental factors could lead to development of macrostomia, but it is usually difficult to single out specific etiological factor. Our patient had negative familial history of facial clefts, of medication, illnesses or trauma during pregnancy. Although, the mother had still birth of her first child but nutritional deficiencies or any history of medication in the pregnancy could not be established. Child had 12 years old brother who was normal in every aspect.

Surgical reconstruction is the mainstay of the management of the defects. Many procedures are described like cutaneous Z-plasty,^2^ W-plasty, commissuroplasty by vermilion square flap and straight line closure^12^ and two triangular flaps^8^ and advancement of oral commissure using a composite flap^13^ are common methods.

Initial workers used Z-plasty to close transverse facial cleft^10,14^ but later on it was noticed that the Z-plasty left a more visible scar. This drawback of Z-plasty lead to development of straight line closure.^15^ Kawai described a technique to correct macrostomia with a simple straight line incision and incorporation of a small triangular flap to achieve proper positioning of the commissure with minimal visible scar.^16^ Eguchi^8^ reported vermilion square flap surgical technique that combines a lower lip mucocutaneous vermilion border flap with a lazy W-plasty to ensure a natural commissure and cheek skin closure.^8^ This technique was used in 8 patients with satisfactory results.

The technique of two triangular flaps allows achieving all therapeutic goals, formation of symmetric lips and commissures of the mouth, reconstruction of the orbicularis muscle of mouth to restore labial function, and reconstruction of the commissure of the mouth with a natural looking contour. The advantage of this technique is that the position of the commissure of the mouth can be adjusted intraoperatively according to the extent of macrostomia.^9^ All these methods emphasize the importance of restoration of the integrity of cheek and lip muscles.

The point of new commissure must be predetermined with accuracy and preoperative marking of the normal landmarks are very important. For better cosmetic and functional outcome and to change the vermilion border the measurements and observations should be jointly considered and matched. Bauer et al used a technique combines triangular mucosal flaps at the commissure and reconstruction of the oral and buccal musculature, and skin closure using a W-plasty. They emphasized that this techniques results in a less conspicuous scar, prevents the lateral drift of the commissure and yields consistent clinical results.

Accurate repair of orbicularis oris is mandatory since this is the muscle which sets the tone to provide a good shape and contour to the commissure. A small triangular skin flap is raised from lower lip and inserted into the commissure, improves the overlapping of the upper and lower lips.^10^ Some authors have reported good results from a vermilion square flap commissuroplasty and triangular flaps.^8^ Yushimura et al^15^ compared 5 children with Z-plasty and 7 with simple line repair. They found less pleasing appearance with Z-plasty. Mahtar et al^17^ have supported that reconstruction of the integrity of the oral sphincter associated with W-plasty usually gives the best results.

Cases of facial cleft should be operated under naso-endotracheal intubation. This gives way for more critical assessment of new point of commissures not only preopera-tively but immediate postoperatively also. This also avoids reconstruction of orbicularis oris under tension which is possible when nasoendotracheal intubation is done. This repair is significant to achieve normal sphincter like function which is necessary for articulation and mastication.

Bilateral transverse facial cleft remains an uncommon congenital malformation, and are sources of mental agony and psychological stress. But a timely surgical intervention and adequate counseling of the family members is the need of the hour.
